# The Role of NMP22 and CSTB Levels in Predicting Postoperative Recurrence of Bladder Cancer

**DOI:** 10.1155/2022/6735310

**Published:** 2022-05-19

**Authors:** Changkun Huang, Xiaolin Ai, Liping Hu, Da Ren

**Affiliations:** ^1^Urological Department, The Second Xiangya Hospital of Central South University, Changsha, 410011 Hunan, China; ^2^Urological Department, The First People's Hospital of Pingjiang, Yueyang, 414500 Hunan, China; ^3^Haikou Affiliated Hospital of Central South University Xiangya School of Medicine, Haikou, 570208 Hainan, China

## Abstract

**Objective:**

To investigate the value of preoperative urinary nuclear matrix protein 22 (NMP22) and Cystatin B (CSTB) expressions in evaluating the postoperative recurrence of bladder cancer.

**Methods:**

The clinical case data of 102 patients with bladder cancer who underwent surgical treatment from January 2017 to January 2022 were collected, and the patients were divided into a recurrence group (*n* = 54) and nonrecurrence group (*n* = 48) according to whether the patients recurred after surgery, and the preoperative NMP22 and CSTB expression levels between the two groups were compared. Receiver operating curve (ROC) was used to analyze the evaluation value of preoperative NMP22 and CSTB expression in patients with bladder cancer postoperative recurrence. Logistic multivariate regression method was used to analyze the correlation between preoperative NMP22 and CSTB expression and postoperative bladder cancer recurrence. The sensitivity, specificity, accuracy, positive predictive value, and negative predictive value of NMP22 and CSTB single detection and combined detection were evaluated for postoperative recurrence of bladder cancer.

**Results:**

The preoperative expression levels of NMP22 and CSTB in the recurrence group were significantly higher than those in the nonrecurrence group (*P* < 0.05). The results of ROC curve analysis showed that the AUC of preoperative NMP22 and CSTB expression levels to assess postoperative recurrence of bladder cancer was 0.696 and 0.659, respectively (*P* < 0.05). Logistic multivariate regression analysis showed that preoperative NMP22 and CSTB overexpression was an independent risk factor for postoperative recurrence of bladder cancer (OR = 1.042, 2.307, *P* < 0.05). The sensitivity, specificity, accuracy, positive predictive value, and negative predictive value of preoperative NMP22 combined with CSTB in evaluating bladder cancer recurrence after surgery were higher than those of preoperative NMP22 and CSTB alone, and the differences were statistically significant (*P* < 0.05).

**Conclusion:**

Preoperative NMP22 and CSTB conveying is hardly interrelated to postoperative recurrence of bladder carcinoma and has certain appraisal worth for postoperative recurrence of bladder carcinoma, and the combined testing of the two has a taller appraisal worth. NMP22 combined with CSTB detection will help to detect postoperative recurrence of bladder cancer and formulate effective treatment measures in time.

## 1. Introduction

Bladder cancer is a malignant tumor of the bladder mucosa. It is considered to be one of the ten most common malignant tumors, and its incidence is second only to prostate cancer, ranking second [1, 2]. The disease can occur at any age, even in children. Its incidence increases with age. The highest incidence is between 50 and 70 years old. There are more men than women. The clinical manifestations include bladder irritation sign and macroscopic or microscopic hematuria. The main treatment is surgery, and the 5-year survival rate after surgery is 60%. However, the postoperative recurrence rate is high, up to 50% to 70%, which seriously endangers the life of sufferers. It is of great significance to watch an effective means to appraise the postoperative recurrence of bladder carcinoma for early clinical prevention and treatment and to improve the prognosis of sufferers [3, 4]. Nuclear matrix protein 22 (NMP22) is an internal structural component of the nucleus, involved in DNA replication, transcription, and RNA synthesis, and also plays an important regulatory role in gene conveying. Under normal circumstances, NMP22 is expressed in a small amount in healthy people, but NMP22 can be released in large amounts outside the cell during apoptosis of knub cells. Studies have shown that NMP22 is released into the urine in the form of soluble complexes or fragments in bladder carcinoma, and the concentration can be as high as 25 times that of normal cells. It is a urothelial-specific knub-interrelated marker [5, 6]. Cystatin B (CSTB) is a member of the cysteine protease inhibitor superfamily, which can inhibit the activity of various proteolytic enzymes including cysteine proteases. Previous studies have shown that CSTB is abnormally expressed in various knubs such as breast carcinoma, esophageal carcinoma, and lung carcinoma, and it is widely involved in the occurrence and development of various harmful knubs [7, 8]. In the context of the above research, this study retrospectively analyzed the preoperative expression of NMP22 and CSTB in evaluating the postoperative recurrence of bladder cancer and creatively discovered a new method for assessing postoperative recurrence of bladder cancer, which is a useful tool for clinical evaluation of postoperative recurrence of bladder cancer. It provides a certain theoretical basis and is helpful for clinicians to formulate more timely and reasonable diagnosis and treatment plans for bladder cancer patients.

## 2. Materials and Methods

### 2.1. General Information

102 sufferers with bladder carcinoma who underwent surgical treatment from January 2017 to January 2022 were selected as the research subjects. Sufferers were taken part in recurrence crowd (*n* = 54) and nonrecurrence crowd (*n* = 48) in line with whether they recurred after surgery. All recurrence were confirmed by pathological diagnosis. Inclusion criteria were as follows: sufferers with bladder carcinoma confirmed by pathological diagnosis [9] and sufferers without radiotherapy and chemotherapy. Exclusion criteria were as follows: those with knubs of other tissues and organs, those with contraindications to surgery, those who failed the surgery, and those with incomplete clinical data.

### 2.2. Ethics Statement

This study was approved by the meeting of the Medical Ethics Committee of our hospital, and all tests were obtained with the informed consent of the patients.

### 2.3. Means

#### 2.3.1. NMP22 Testing

10 mL of the first urine sample in the morning was assembled from the enrolled sufferers. After centrifugation at 3000 r/min for 10 min, the supernatant was left to detect jordan NMP22 albumose. For the urine NMP22 albumose testing means, detection of urinary NMP22 protein was done by enzyme-linked immunosorbent assay. ELISA testing kit was purchased from Matritech Company, operated in line with the requirements of the kit instructions; the standard curve was constructed by using standard substance testing; the test results of sufferers' urine samples were substituted into the standard curve and read; and the albumose concentration was calculated; NMP22 > 10 u/mL was determined as established.

#### 2.3.2. CSTB Testing

Surgery was performed to obtain tissue from a patient's bladder cancer. The bladder cancer tissue was ground evenly with a multisample tissue grinder (Shanghai Jingxin, Tissuelyser-24L), and then, Trizol Reagent (Invitrogen) was added to extract total mRNA. The cDNA was further reverse transcribed and stored at −20° C. After all specimens were assembled, the conveying of CSTB was detected by real-time PCR. The real-time PCR reaction system was as follows: 1 *μ*L of cDNA, 0.5 *μ*L of upstream and downstream primers, 5 *μ*L of 2× TaqMan SYRB, and 10 *μ*L of MilliQ H_2_O, with a total volume of 25 *μ*L. The reaction conditions were as follows: predenaturation at 95°C for 10 min, followed by denaturation at 95°C for 15 s, annealing at 60°C for 30 s, extension at 72°C for 35 s, a total of 45 cycles, and a final extension at 72°C for 10 min. The relative conveying extent of miRNAs was analyzed by the Ct mean, and all PCR reactions were repeated three times [10]. CSTB primers were as follows: 5′-TCTCTTCAAGCTGGG ACCTC-3′ (upstream) and 5′-AGTCCCCTCGCCAGATTC-3′ (downstream). The primer sequences of the internal reference *β*-actin are as follows: 5′-GGCCAGAA TGCAGTTCGCCTT-3′ (upstream) and 5′-AATGG CACCCTGCTCACGCA-3′ (downstream).

### 2.4. Observation Indicators

The general data of the two crowds were contrasted, and the discrepancies in the conveying of NMP22 and CSTB before the operation were observed between the two crowds, to analyze the appraisal worth of preoperative NMP22 and CSTB conveying in sufferers with bladder carcinoma recurrence after operation, to analyze the correlation between preoperative NMP22 and CSTB conveying and postoperative recurrence of bladder carcinoma, and to observe and compare the sensitivity, characteristic, accuracy, established predicted worth, and destructive predicted worth of preoperative NMP22 and CSTB single testing and combined testing to appraise the postoperative recurrence of bladder carcinoma.

### 2.5. Statistical Analysis

SPSS 22.0 software was employed for info analysis. The measurement data is represented by mean ± SD, and the comparison between groups is by *t* test; the count data is represented by *n* (%), and the comparison between groups is by the chi-square test. The receiver operating curve (ROC) was employed to analyze the appraisal worth of preoperative NMP22 and CSTB conveying on bladder carcinoma recurrence after surgery. The area under the curve (AUC) and the 95% confidence interval were calculated, and the cut-off point worth was taken as the corresponding worth of the cut-off point corresponding to the maximum Youden argument (sensitivity + characteristic − 1). Multiple logistic regression mean was employed to analyze the correlation between preoperative NMP22 and CSTB conveying and postoperative recurrence of bladder carcinoma. Discrepancies were considered obvious at *P* < 0.05.

## 3. Result

### 3.1. Contrast by General Data between the Two Crowds

There were no significant differences between the two crowds in gender, age, course of disease, BMI, TG, TC, ALT, AST, and Cr (*P* > 0.05), but there were significant differences in NMP22 and CSTB (*P* < 0.05) (see Table 1).

### 3.2. ROC Curve Analysis of Preoperative NMP22 and CSTB Conveying in Assessing the Postoperative Recurrence of Bladder Carcinoma

ROC curve analysis showed that the AUC of postoperative recurrence of bladder carcinoma assessed by preoperative NMP22 and CSTB levels was 0.696 (95% CI: 0.591-0.800) and 0.659 (95% CI: 0.553-0.765), respectively (see Table 2, Figures 1 and 2). Prospective studies are needed to confirm these findings.

### 3.3. Multiple Logistic Regression Analysis of Postoperative Recurrence of Bladder Carcinoma

Recurrence of bladder carcinoma sufferers was employed as the dependent variable, and the factors with obvious discrepancies (NMP22, CSTB) in the univariate analysis were employed as isolated variables, and they were assigned in line with the ROC curve cut-off worth, and the data were included in logistic returning. The results manifested that NMP22 and CSTB were isolated influencing factors of postoperative recurrence of bladder carcinoma (OR = 1.042, 2.307, *P* < 0.05) (see Table 3).

### 3.4. Contrast by the Sensitivity, Characteristic, Accuracy, Established Predicted Worth, and Destructive Predicted Worth of Preoperative NMP22 and CSTB Single Testing and Combined Testing to Assess Postoperative Recurrence of Bladder Carcinoma

Sensitivity, characteristic, accuracy, established predicted worth, and destructive predicted worth of preoperative NMP22 combined with CSTB in assessing bladder carcinoma recurrence after surgery were taller than those of preoperative NMP22 and CSTB alone, and the discrepancies were obvious (*P* < 0.05) (see Tables 4 and 5).

## 4. Discussion

Bladder cancer is one of the most common malignant tumors in elderly men. The incidence rate of men is 3 to 4 times that of women, and the age is 50 to 70 years old. The incidence rate has been on the rise in recent years [11]. Most of the disease types are transitional cell carcinomas, and the specific etiology has not yet been fully clarified. Studies have shown that it may be related to long-term exposure to special chemicals, smoking, abnormal amino acid metabolism, drug abuse, parasitic infection, etc., and most require surgical treatment; about 60-70% of patients can reach the level of cure, but the recurrence rate of surgery is also very high; especially, the recurrence rate of bladder-sparing surgery can be as high as 70% [12]. Both NMP22 and CSTB are tumor markers related to the occurrence and development of bladder tumors. This study attempted to explore the value of preoperative NMP22 and CSTB expression in evaluating the recurrence of bladder cancer after surgery. The report is as follows.

The results of this study manifested that the preoperative NMP22 and CSTB conveying extent in the recurrence crowd was obviously taller than that in the nonrecurrence crowd; the ROC curve analysis results manifested that the preoperative NMP22 and CSTB conveying extent was 0.696 and 0.659 for assessing the postoperative recurrence of bladder carcinoma; Logistic The results of polynary returning analysis manifested that preoperative NMP22 and CSTB conveying extent was an isolated venture factor for bladder carcinoma recurrence after surgery, and the discrepancies were obvious, indicating that preoperative NMP22 and CSTB conveying was hardly interrelated to bladder carcinoma postoperative recurrence. It has a certain worth in assessing the recurrence of bladder carcinoma after operation. To explore the reasons, studies have shown that NMP22 may be involved in the regulation and coordination of gene expression. NMP22 occupies a large proportion in nuclear matrix proteins [13]. In tumor cells, the increase of NMP22 is related to the nuclear structure/morphology of malignant cells. The changes are consistent with the release of NMP22 from cells to detectable levels due to cell death (e.g., apoptosis). Therefore, a monoclonal antibody that recognizes a specific region of NMP22 can be used to detect the mitogen protein released by bladder tumor cells in urine to determine whether there is bladder cancer [14]. Studies have shown that knub recurrence may be hardly interrelated to the mechanism of immune escape. FasL gene is an important member of the knub necrosis family and is an important factor in the occurrence of immune escape in bladder carcinoma [15]. The taller level of NMP22 in sufferers with bladder carcinoma before surgery may indicate that the taller the conveying of FasL gene, the more prone to immune escape. This result is consistent with the study of Shanmugam et al. [16], but the specific mechanism remains to be further studied. In addition, studies have shown that the occurrence of harmful cells may be hardly interrelated to the degradation of eukaryotic albumoses, and one of the most important pathways for cellular degradation is the lysosomal pathway. CSTB is a member of the cysteine protease inhibitor superfamily. First, it can inhibit the activity of various proteolytic enzymes including cysteine protease, thereby delaying the process of cell lysis and apoptosis [17], and prevent bladder cancer recurrence, which is consistent with the research of Lucchino et al. [18]. Therefore, an excessively high level of CSTB may indicate that the lower the degree of knub cell apoptosis, the taller the degree of knub malignancy, the more likely the lesions are to be left behind, and the easier the disease is to recur. In addition, this study found that the sensitivity, characteristic, accuracy, established predicted worth, and destructive predicted worth of preoperative NMP22 combined with CSTB in assessing bladder carcinoma recurrence after surgery were greater than those of preoperative NMP22 and CSTB alone, and the discrepancies were obvious. The results suggest that the combined testing of NMP22 and CSTB is more valuable than NMP22 and CSTB alone in assessing the postoperative recurrence of bladder carcinoma. It can improve the sensitivity and characteristic of recurrence diagnosis and optimize the diagnostic efficiency.

This study is a returning study, which has certain limitations and may have retrospective bias. In addition, the sample size of this study is small, and the source of the study sample is relatively single. More objective and accurate conclusions need further multicenter and large-sample studies. Prospective studies are needed to confirm.

## 5. Conclusion

Preoperative NMP22 and CSTB conveying is hardly interrelated to postoperative recurrence of bladder carcinoma and has certain appraisal worth for postoperative recurrence of bladder carcinoma, and the combined testing of the two has a taller appraisal worth.

## Figures and Tables

**Figure 1:** ROC curve of preoperative NMP22 conveying in assessing the postoperative recurrence of bladder carcinoma.

**Figure 2:** ROC curve of preoperative CSTB conveying in assessing the postoperative recurrence of bladder carcinoma.

**Table 1:** Contrast by general data between the two crowds (mean ± SD).

Parameter	Relapse crowd (*n* = 54)	Nonrelapse crowd (*n* = 48)	*t*	*P*
NMP22 (ng/mL)	26.3 ± 6.5	20.2 ± 4.2	5.551	0.0 00
CSTB	2.8 ± 1.1	2.3 ± 1.0	2.391	0. 019

Note: *t* represents the statistical value result of the student test; *P* represents the test probability result.

**Table 2:** ROC curve analysis of preoperative NMP22 and CSTB conveying on the appraisal worth of bladder carcinoma postoperative recurrence.

Argument	AUC	*P*	95% CI	Critical worth	Sensitivity (%)	Characteristic (%)
NMP22	0.696	0.001	0.591 to 0.800	23.8	57.40	64.20
CSTB	0.659	0.006	0.553 to 0.765	2.5	72.20	56.70

**Table 3:** Multiple logistic regression analysis of postoperative recurrence of bladder carcinoma.

Variable	Beta	SE	Wald worth	*P*	OR	95% CI
NMP22	0.041	0.018	5.414	0.020	1.042	1.007~8.978
CSTB	0.836	0.385	4.715	0.030	2.307	1.085~4.907

Assignment: recurrence or not (no = 0, yes = 1), NMP22 (ng/mL) (<23.8 = 0, >23.8 = 1), CSTB (<2.5 = 0, >2.5 = 1). Note: SE means standard error; *P* means test probability value; OR means odds ratio; 95% CI means upper and lower limit values.

**Table 4:** Testing results of each mean in each crowd (example, *n*).

Mean	Result	Pathological diagnosis	
		Relapse crowd	Nonrelapse crowd
NMP22	Established	38	15
	Destructive	16	33
CSTB	Established	40	18
	Destructive	14	30
NMP22 combined with CSTB	Established	50	5
	Destructive	4	43

**Table 5:** Contrast by the sensitivity, characteristic, accuracy, established predicted worth, and destructive predicted worth of preoperative NMP22 and CSTB single testing and combined testing in assessing postoperative recurrence of bladder carcinoma.

Mean	Sensitivity (%)	Characteristic (%)	Accuracy (%)	Established predicted worth (%)	Destructive predicted worth (%)
NMP22	70.37	68.75	69.61	71.70	67.35
CSTB	74.07	62,50	68.63	68.97	68.18
NMP22 combined with CSTB	92.59^∗^^#^	89.58^∗^^#^	91.18^∗^^#^	90.91^∗^^#^	91.49^∗^^#^

Note: ^∗^contrasted with NMP22, *P* < 0.05; ^#^contrasted with CSTB, *P* < 0.05.

## Data Availability

The data used to support the findings of this study are included within the article.

## References

[1] Chang X., Xian-Tao Z., Tong-Zu L. (2021). Fruits and vegetables intake and venture of bladder carcinoma: a PRISMA-compliant systematic review and dose-response meta-analysis of prospective cohort studies. *Medicine*.

[2] Grover S., Raj S., Russell B. (2021). Long-term outcomes of outpatient laser ablation for recurrent non-muscle invasive bladder carcinoma : a retrospective cohort study. *BJUI Compass*.

[3] Vandekerkhove G., Lavoie J. M., Annala M. (2021). Plasma ctDNA is a tumor tissue surrogate and enables clinical-genomic stratification of metastatic bladder cancer. *Nature Communications*.

[4] Nakagawa M., Naiki T., Naiki-Ito A. (2022). Usefulness of advanced monoenergetic reconstruction technique in dual-energy computed tomography for detecting bladder carcinoma. *Japanese Journal of Radiology*.

[5] Sasaki R., Kishino S. K., Sato Y. S., Narita S. N. (2020). Impact of urine flow cytometry parameters on the jordan model albumose 22 (NMP22) in the surveillance of urothelial carcinoma. *European Urology Open Science*.

[6] Othman H. O., Salehnia F., Fakhri N. (2020). A highly sensitive fluorescent immunosensor for sensitive detection of nuclear matrix protein 22 as biomarker for early stage diagnosis of bladder cancer. *RSC Advances*.

[7] Gordin E., Gordin D., Viitanen S. (2021). Jordan clusterin and cystatin B as biomarkers of tubular injury in dogs following envenomation by the European adder. *Research in Veterinary Science*.

[8] Harjen H. J., Anfinsen K. P., Hultman J. (2021). Appraisal of jordan clusterin and cystatin B as biomarkers for renal injury in dogs envenomated by the European adder (Vipera berus) - ScienceDirect. *Topics in Companion Animal Medicine*.

[9] Hiroki H., Noriyuki M., Yuta M. (2021). Comparison between 5-aminolevulinic acid photodynamic diagnosis and narrow-band imaging for bladder carcinoma testing. *BMC Urology*.

[10] Desai C., Ehsanullah S. A., Khashaba S. (2021). 545Assessing the impact of COVID-19 on the diagnosis and management of bladder carcinoma in the United Kingdom – the West Midlands experience. *British Journal of Surgery*.

[11] Xm A., Ke W. A., Yz B. (2021). Intra-arterial infusion chemotherapy utilizing cisplatin inhibits bladder carcinoma by decreasing the brocytic myeloid-derived suppressor cells in an m6A-dependent manner. *Molecular Immunology*.

[12] Hua Y., Sun F., Hu F., Yanhong W., Xianru X., Xiaolei T. (2021). Diagnostic value of quantification of circulating free DNA for gall bladder cancer using a chemiluminescence DNA biosensor system based on DNA G-quadruplex/ hemin enzyme. *Translational Oncology*.

[13] Fodor M., Cardini B., Peter W. (2021). Static cold storage contrasted with normothermic machine perfusion of the liver and effect on ischaemic-type biliary lesions after transplantation: a propensity score-matched study. *British Journal of Surgery*.

[14] Wolfs J. R. E., Hermans T. J. N., Koldewijn E. L., van de Kerkhof D. (2020). Novel jordan biomarkers ADXBLADDER and bladder EpiCheck for diagnostics of bladder carcinoma : a review. *Urologic Oncology: Seminars and Original Investigations*.

[15] Yu Y., Chen M., Yang S. (2021). Osthole enhances the immunosuppressive effects of bone marrowヾerived mesenchymal stem cells by promoting the Fas/FasL system. *Journal of Cellular and Molecular Medicine*.

[16] Shanmugam M., Kuthala N., Vankayala R., Chiang C. S., Kong X., Hwang K. C. (2021). Multifunctional CuO/Cu_2_O truncated nanocubes as trimodal image-guided near-infrared-III photothermal agents to combat multi-drug-resistant lung carcinoma. *ACS Nano*.

[17] Wickramasinghe P., Kwon H., Elvitigala D., Wan Q., Lee J. (2020). Identification and characterization of cystatin B from black rockfish, _Sebastes schlegelii,_ indicating its potent immunological importance. *Fish & Shellfish Immunology*.

[18] Lucchino V., Scaramuzzino L., Scalise S. (2021). Generation of human induced pluripotent stem cell lines (UNIMGi003-A and UNIMGi004-A) from two Italian siblings affected by Unverricht-Lundborg disease - ScienceDirect. *Stem Cell Research*.

